The article "Ellagic Acid: A Review on Its Natural Sources, Chemical Stability, and Therapeutic Potential" was retracted in 2024. Reasons: signs of a paper mill; compromised peer review; unreliable results or conclusions.

# Ellagic Acid: A Review on Its Natural Sources, Chemical Stability, and Therapeutic Potential

**DOI:** 10.1155/2022/3848084

**Published:** 2022-02-21

**Authors:** Javad Sharifi-Rad, Cristina Quispe, Carla Marina Salgado Castillo, Rodrigo Caroca, Marco A. Lazo-Vélez, Halyna Antonyak, Alexandr Polishchuk, Roman Lysiuk, Petro Oliinyk, Luigi De Masi, Paola Bontempo, Miquel Martorell, Sevgi Durna Daştan, Daniela Rigano, Michael Wink, William C. Cho

**Affiliations:** ^1^Facultad de Medicina, Universidad del Azuay, Cuenca, Ecuador; ^2^Facultad de Ciencias de la Salud, Universidad Arturo Prat, Avda. Arturo Prat 2120, Iquique 1110939, Chile; ^3^Biotechnology and Genetic Engineering Group, Science and Technology Faculty, Universidad del Azuay, Av. 24 de Mayo 7-77, Cuenca, Ecuador; ^4^Universidad del Azuay, Grupos Estratégicos de Investigación en Ciencia y Tecnología de Alimentos y Nutrición Industrial (GEICA-UDA), Av. 24 de Mayo 7-77, Apartado 01.01.981, Cuenca, Ecuador; ^5^Ivan Franko National University of Lviv, Lviv, Ukraine; ^6^Danylo Halytsky Lviv National Medical University, Lviv, Ukraine; ^7^National Research Council (CNR), Institute of Biosciences and Bioresources (IBBR), Via Università 133, 80055 Portici, Naples, Italy; ^8^Department of Precision Medicine, University of Campania “Luigi Vanvitelli”, Via L. De Crecchio 7, 80138 Naples, Italy; ^9^Department of Nutrition and Dietetics, Faculty of Pharmacy, and Centre for Healthy Living, University of Concepción, 4070386 Concepción, Chile; ^10^Department of Biology, Faculty of Science, Sivas Cumhuriyet University, 58140 Sivas, Turkey; ^11^Beekeeping Development Application and Research Center, Sivas Cumhuriyet University, 58140 Sivas, Turkey; ^12^Department of Pharmacy, University of Naples “Federico II”, Via D. Montesano, 49 80131 Naples, Italy; ^13^Heidelberg University, Institute of Pharmacy and Molecular Biotechnology, INF 329, D-69120 Heidelberg, Germany; ^14^Department of Clinical Oncology, Queen Elizabeth Hospital, Kowloon, Hong Kong

## Abstract

Ellagic acid (EA) is a bioactive polyphenolic compound naturally occurring as secondary metabolite in many plant taxa. EA content is considerable in pomegranate (*Punica granatum* L.) and in wood and bark of some tree species. Structurally, EA is a dilactone of hexahydroxydiphenic acid (HHDP), a dimeric gallic acid derivative, produced mainly by hydrolysis of ellagitannins, a widely distributed group of secondary metabolites. EA is attracting attention due to its antioxidant, anti-inflammatory, antimutagenic, and antiproliferative properties. EA displayed pharmacological effects in various *in vitro* and *in vivo* model systems. Furthermore, EA has also been well documented for its antiallergic, antiatherosclerotic, cardioprotective, hepatoprotective, nephroprotective, and neuroprotective properties. This review reports on the health-promoting effects of EA, along with possible mechanisms of its action in maintaining the health status, by summarizing the literature related to the therapeutic potential of this polyphenolic in the treatment of several human diseases.

The article "Ellagic Acid: A Review on Its Natural Sources, Chemical Stability, and Therapeutic Potential" was retracted in 2024. Reasons: signs of a paper mill; compromised peer review; unreliable results or conclusions.

## 1. Introduction

Ellagic acid (EA) was first discovered in 1831 by the French chemist and pharmacist Henri Braconnot who named it “acide ellagique” from the reverse-read word “galle” [1]. However, the presence of this substance in plants was not clearly understood until the early 20th century, when it was prepared from various plant sources such as oak bark, valonea, pomegranate (*Punica granatum* L.), divi-divi (*Caesalpinia coriaria* (Jacq.) Willd.), myrobalan (*Terminalia catappa* L.), and algarrobilla (*Prosopis humilis* Hook.) [1]. At present, EA is known as a naturally occurring bioactive and pharmacologically active polyphenolic compound that is abundant in many taxonomically diverse plant groups, mainly among eudicotyledons [2–4]. Structurally, EA constitutes a dilactone of hexahydroxydiphenic acid (HHDP), which can be considered a dimeric gallic acid derivative. EA is produced in plants mainly via hydrolysis of ellagitannins, a widely distributed group of plant secondary metabolites [5–10]. Along with free EA, plants capable of synthesizing ellagitannins contain a range of EA derivatives with varying structural complexity, which arise as a result of methylation, methoxylation, glycosylation, and glucuronidation of its molecule [11–14]. Ellagitannins, hydrolysable derivatives of EA, can release it in a free form in the human gastrointestinal tract after consuming plant-based foods.

In recent decades, EA is attracting great attention due to its pronounced antioxidant [15–23], anti-inflammatory [24–29], antimutagenic [30–33], and antiproliferative properties [34–39] and its therapeutic potential in the treatment of several human diseases. Numerous studies have shown that EA may be involved in regulating a spectrum of cellular signaling pathways to prevent, mitigate, or slow down the progression of chronic disorders, including cardiovascular [40–43] and neurodegenerative diseases [44–47], diabetes [48–51], and cancer [38, 52–54]. This compound has also been shown to exhibit neuroprotective [55–59], hepatoprotective [60–68], nephroprotective [69, 70], cardioprotective [71–73], antifibrotic [74], antiatherosclerotic [75, 76], antiallergic [77–79], antinociceptive [80–82], antiestrogenic [83], skin-protecting [84–87], wound-healing [88–90], osteogenic [91–93], antimicrobial [20, 37, 94], antiviral [19, 95–97], and antiparasitic [98–100] effects. In addition, EA has shown a protective effect against the toxicity of metals and metalloids [101–106], organic xenobiotics [107–111], and natural toxins [112–114]. There is also evidence of a positive therapeutic effect of the combination of EA with other antioxidants, including selenium (in the form of selenomethionine) [115], known for its multiple biological activities and therapeutic potential [116–120]. This review is aimed to reporting the health-promoting effects of EA, along with possible mechanisms of its action in maintaining the health status, by summarizing the literature related to the therapeutic potential of this polyphenolic in the treatment of several human diseases.

The article "Ellagic Acid: A Review on Its Natural Sources, Chemical Stability, and Therapeutic Potential" was retracted in 2024. Reasons: signs of a paper mill; compromised peer review; unreliable results or conclusions.

## 2. Chemical Properties and Natural Sources of EA

EA is a thermostable molecule with a melting point of 350°C, a molecular weight of 302.19 g/mol, almost insoluble in water and sparingly soluble in alcohol [1, 121]. From a chemical point of view, EA is identified as 2,3,7,8-tetrahydroxy-chromeno [5,4,3-*cde*]chromene-5,10-dione.

EA has the properties of an amphiphilic molecule; structurally, it consists of a planar biphenyl lipophilic moiety bridged by two lactone rings and possessing four hydroxyl groups, which together with lactone groups form a hydrophilic moiety [122]. The hydrophilic part of the EA molecule plays an important role in its biological activity due to the presence of both hydrogen bonding acceptor (lactone) and donor (–OH) sites (phenolic hydroxyl groups which can dissociate under physiological conditions to negatively charged phenolate ions) [123].

In plant cells, EA is contained in free and covalently bound forms, including EA glycosides and ellagitannins, each having different chemical reactivity, solubility, and bioavailability [124–126]. To date, a broad spectrum of ellagitannins and EA glycosides have been isolated and studied from various plant species. EA glycosides contain sugar residues such as glucose, arabinose, xylose, or rhamnose [12]. Both ellagitannins and EA glycosides are hydrolysable compounds and can release EA upon hydrolysis both in plants and in the gastrointestinal tract of humans and herbivore animals.

Due to a wide range of biological effects of EA, edible plants containing this phytochemical and its hydrolyzable derivatives, mainly ellagitannins, are a valuable source of EA for humans and belong to functional foods that promote health and may reduce the risk of disease [127, 128]. Many species of medicinal plants used in traditional medicine around the world, including Traditional Chinese Medicine and Ayurveda, have been found to contain EA and ellagitannins [63, 97, 129–134]. EA is currently used in the pharmaceutical and cosmetics industries. Consequently, various plant species are now being studied for EA content in order to find novel sources of EA in human nutrition, as well as sources of raw materials for the preparation of functional nutritional supplements and nutraceuticals.

The article "Ellagic Acid: A Review on Its Natural Sources, Chemical Stability, and Therapeutic Potential" was retracted in 2024. Reasons: signs of a paper mill; compromised peer review; unreliable results or conclusions.

Although ellagitannins and EA derivatives are widespread in the plant kingdom, only a limited number of plant species have been reported with substantially high levels of these phytochemicals and, consequently, as rich natural sources of EA in human nutrition. In particular, high concentrations of both ellagitannins and EA are found in fruits (especially berries), in nut kernels, and, in some cases, in other parts of the plant. Considering the level of conversion of ellagitannins to EA, the highest concentrations of EA are found in fruits of plants of the genus *Rubus* (raspberry, cloudberry, arctic bramble, blackberry, and boysenberry), strawberry (*Fragaria × ananassa* (Duchesne ex Weston) Duchesne ex Rozier), pomegranate, muscadine grape (*Vitis rotundifolia* Michx.), and tropical fruits such as camu-camu (*Myrciaria dubia* (Kunth) McVaugh); walnuts (*Juglans* spp.) and pecan (*Carya illinoinensis* (Wangenh.) K.Koch) have also relatively high EA content (Table 1) [4, 36, 121, 126, 135–139]. These plants are the main sources of EA in the human diet. Other sources of EA in human nutrition are juices, jams, and other processed products of ellagitannin-containing plants in the food industry. In particular, pomegranate juice (PJ) may contain a total EA concentration of 811 mg/L [140] and higher [141] due to the high content of ellagitannins in *P. granatum* fruits.

It should be noted that despite the fact that early studies did not show the presence of EA in plants of the Fabaceae family [11, 142], there is now evidence of relatively high levels of this phytochemical in several sprouted legumes, such as sprouted adzuki bean (*Vigna angularis*), some varieties of bean (*Phaseolus vulgaris* L.), cowpea (*Vigna unguiculata* (L.) Walp.), pea (*Pisum sativum* L.), and soybean (*Glycine max* (L.) Merr.) [143]. Sprouted soybeans have been found to have a considerably higher EA content than other sprouted legumes (45.6–48.9 and 8.96–18.3 mg/100 g dry weight, respectively) [143].

The ratio between free and bound forms of EA in plant tissues varies considerably depending on the plant species; however, the proportion of unbound EA may also depend on the method chosen for determination. According to some authors, free EA makes up only a small part of the total EA pool in plants [144–146], while others suggest that its portion can reach and even exceed 50% of the total content [147, 148]. Interestingly, in the fruits of *Terminalia ferdinandiana* Exell, a native Australian plant known as the Kakadu plum, EA was found to be mostly free form, with a percentage reaching 70.6% of the total EA pool [125]. By contrast, the percentage of free EA in strawberries, as shown by the same study, reaches 7.4% of its total content [125].

The article "Ellagic Acid: A Review on Its Natural Sources, Chemical Stability, and Therapeutic Potential" was retracted in 2024. Reasons: signs of a paper mill; compromised peer review; unreliable results or conclusions.

It has been shown that storing and freezing fruits, as well as processing them for the production of beverages and jams, may have different effects on the content of EA. In particular, industrial processing of pomegranates for juice production increases the concentration of EA in juices; at the same time, juice prepared from frozen fruits contains two times less of this compound than juice prepared from fresh fruits [152]. Significant increases in the content of EA (2–3 times) were observed during the processing of raspberries for jam production and during 1–6 months of storage of raspberry jam [144]. However, processing strawberries for jam production has been shown to reduce total EA content by 20% [153].

Some tree species have a particularly high EA content in wood and bark, such as *Quercus* spp., *Eucalyptus* spp., and *Castanea* spp. [154–157]. Consequently, by-products of the forestry and wood-processing industries (as well as by-products of juice production such as pomegranate husk) are a potential source of industrial production for EA [149].

## 3. Ellagitannins as a Source of Ellagic Acid

### 3.1. General Characteristic and Biosynthesis of Ellagitannins in Plants

Ellagitannins represent one of the most diverse groups of plant phenolics and encompass over 1,000 identified natural bioactive compounds [8]. These phytochemicals have a tart taste and pronounced astringent properties and are capable of forming complexes with proteins and polysaccharides [158]. Ellagitannins are located in the vacuoles and cytoplasm of plant cells and play an important protective role in natural growth conditions, providing a chemical defense against infection by microbial pathogens and herbivore attack [159].

By their chemical nature, ellagitannins are hydrolyzable tannins and constitute the largest group among them [8]. These compounds are found in the form of (1) monomers, (2) *C*-glycosidic ellagitannins with an open-chain glucose moiety, (3) oligomers, and (4) complex tannins; the molecular weight of ellagitannins ranges from 300 to 20,000 Da [7, 160]. A characteristic feature of the chemical structure of all ellagitannins is the presence of at least one HHDP unit, which is esterified to a polyol, typically *β*-D-glucose. The HHDP moiety arises due to the oxidative C–C bond formation between neighboring galloyl residues within the ellagitannin structure. Another group of hydrolyzable tannins is represented by gallotannins (polygalloyl esters of glucose or other polyol carbohydrate), which have a simpler structure and more restricted distribution in nature than ellagitannins [160, 161]. A molecular precursor of both gallotannins and ellagitannins in plants is gallic acid (3,4,5-trihydroxybenzoic acid), and the initial stages of biosynthesis are common to both of these groups of phytochemicals [158].

The article "Ellagic Acid: A Review on Its Natural Sources, Chemical Stability, and Therapeutic Potential" was retracted in 2024. Reasons: signs of a paper mill; compromised peer review; unreliable results or conclusions.

The pathway for the synthesis of a simple ellagitannin molecule in plants includes several stages, as follows: (1) the formation of gallic acid via the shikimate pathway with 3-dehydroshikimic acid as an intermediate [162], (2) the enzymatic formation of 1-*O*-galloyl-*β*-D-glucose and its sequential galloylation to generate 1,2,3,4,6,-penta-*O*-galloyl-*β*-D-glucose (the central molecule in the biosynthesis of all hydrolyzable tannins), and (3) the oxidative coupling of two neighboring galloyl groups to form the HHDP moiety [163]. Following the formation of the first HHDP unit, the formation of the second HHDP unit can occur, as well as the subsequent cleavage of HHDP or galloyl units from the rest of the molecule [8].

The diversity of the structure of simple ellagitannins is mainly associated with various possible variants of the formation of linkages between the HHDP group(s) and the glucose moiety, as well as with the occurrence of axial chirality on the HHDP group. In this way, the *S*- or *R*-configurations arise depending on bond formation at the *O*-2,*O*-3- and/or *O*-4,*O*-6-positions in the glucopyranose core or at the *O*-3,*O*-6-positions, respectively [8, 164]. An additional one or two galloyl groups can bind to the HHDP moiety via oxidative coupling, resulting in the formation of nonahydroxytriphenoyl (NHTP) and gallagyl groups, respectively [164]. Variations in ellagitannin structure also arise due to formation of C–O bonds between the galloyl and HHDP units, as well as due to oxidation of the HHDP group. As a result of intermolecular oxidative processes, other groups such as sanguisorboyl, tergalloyl, valoneoyl, dehydrohexahydroxydiphenoyl (DHHDP), and chebuloyl, are formed in ellagitannin structure [8]. Various monomeric forms of ellagitannins often bind together to form oligomers, which significantly increases their structural diversity. The oligomerization process results in decreased solubility and/or covalent attachment of ellagitannins to cell wall components [165]. Ellagitannins can also form complex structures (complex tannins) in which the ellagitannin unit is linked by a glycosidic bond to the catechin unit [160].

The article "Ellagic Acid: A Review on Its Natural Sources, Chemical Stability, and Therapeutic Potential" was retracted in 2024. Reasons: signs of a paper mill; compromised peer review; unreliable results or conclusions.

### 3.2. Distribution of Ellagitannins in Plants

Ellagitannins are synthesized in eudicotyledons, mainly in polypetalous plants, and have been detected in genera of many plant families, including Anacardiaceae, Betulaceae, Combretaceae, Cornaceae, Euphorbiaceae, Fabaceae, Fagaceae, Ebenaceae, Geraniaceae, Juglandaceae, Lythraceae, Melastomataceae, Myrtaceae, Nymphaeaceae, Onagraceae, Paeoniaceae, Phyllanthaceae, Polygonaceae, Punicaceae, Rosaceae, Sapindaceae, Saxifragaceae, Staphyleaceae, Theaceae, Tamaricaceae, and Vitaceae [5, 7, 145, 166–172]. Among these plants are woody, shrub, and herbaceous species, many of which are traditionally used in medical practice in various countries.

In plants of the genus *Rubus* (raspberry, blackberry, and cloudberry), ellagitannins have been shown to represent the major group of phenolic compounds, while ellagitannins in *Fragaria* spp. (strawberry) are the second largest group of phenolics after anthocyanins [173]. The main ellagitannins synthesized in *Rubus* spp. are sanguine H-6 and lambertianine C [174, 175], which are also found as minor components in *Fragaria* spp. [176]. In strawberry, the main ellagitannin is agrimoniin, which has a structure of *α*-galloyl-HHPP-glucose dimmer [176, 177]. Typical ellagitannin of pomegranate (*P. granatum*) is punicalagin, while walnut (*Juglans regia* L.) and pecan (*C. illinoinensis*) contain pedunculagin as the main ellagitannin [178].

Ellagitannins can be found in virtually all parts of plants capable of synthesizing these compounds, including roots, leaves, bark, wood, galls, fruits, and seeds. In many plant species, these compounds occur simultaneously with gallotannins or other groups of tannins. In particular, in pomegranate, ellagitannins are mainly found in the pericarp, bark, seeds, and flowers, while gallotannins are contained mostly in leaves [179]; species of the genera *Caesalpinia*, *Quercus*, *Myroxylon*, *Rhus*, *Prosopis*, and others also contain both ellagitannins and gallotannins [167]; young oak leaves contain mostly ellagitannins, and oak bark yields a mixture of ellagitannins and condensed tannins (proanthocyanidins) [154]. Ellagitannins are also found in oak-aged wines as a result of their leakage from the oak barrel into the wine [178].

In oak wood, ellagitannins can represent up to 10% of the dry material [180]. In pomegranate, the concentration of its main ellagitannin, punicalagin, ranges from 11 to 20 g/kg in the mesocarp and peel and from 4 to 565 mg/L in juice [181]. Berries such as raspberry and cloudberry have been shown to contain ellagitannins at concentrations of up to 330 mg/100 g of fresh weight (FW), while rose hips and different varieties of strawberry contain, respectively, 110 and around 70 mg ellagitannins per 100 g FW; the content of ellagitannins in jams is 22–32% of those in unprocessed berries [145].

The article "Ellagic Acid: A Review on Its Natural Sources, Chemical Stability, and Therapeutic Potential" was retracted in 2024. Reasons: signs of a paper mill; compromised peer review; unreliable results or conclusions.

### 3.3. Decomposition of Ellagitannins

Ellagitannins can decompose to yield EA enzymatically or under acidic and alkaline conditions [182, 183]. Enzymatic hydrolysis of ellagitannins, which occurs naturally in plants, as well as their enzymatic decomposition in the gastrointestinal tract of humans and animals, when ellagitannin-containing plants are consumed, leads to the formation of EA. In addition, a range of microorganisms can degrade these compounds under natural and laboratory conditions due to possessing enzymes breaking the ester bonds between the HHDP groups and glucose [168, 184, 185].

Current evidence based on laboratory studies of the enzymatic degradation of ellagitannins to form EA suggests that two alternative enzymes could potentially be involved in this process. One of these may be tannase (tannin acyl hydrolase, EC 3.1.1.20), an enzyme found in plants and microorganisms, which is known to catalyze the breakdown of hydrolyzable tannins, including ellagitannins [186, 187] and ellagitannin acyl hydrolase (ellagitannase), an inducible enzyme that has been reported to be produced by micromycetic fungi [184]. However, recent studies have demonstrated that EA release is strongly associated to ellagitannase activity [184, 185, 188]. It has been shown that ellagitannase catalyzes the hydrolysis of ester bonds between glucose and the HHDP group of ellagitannins, giving rise to HHDP; the latter undergoes rapid lactonization with the formation of EA (Figure 1) [184]. Unlike tannase, ellagitannase does not act on gallotannins [189].

### 3.4. Biological Effects of Ellagitannins

Numerous data suggest that ellagitannins exhibit a wide range of biological and clinically relevant activities and have the potential for health promotion and medical applications, including cancer prevention and treatment [8, 190–197].

However, due to the complexity of their structure, most of the ellagitannins from various sources are not absorbed in the human gastrointestinal system. Therefore, the strong bioactivity of dietary ellagitannins can be explained by their ability to be hydrolyzed in the digestive system, primarily to EA and other smaller polyphenols, and also to produce biologically active metabolites *in vivo*. At the same time, the health-promoting effects of ellagitannins are also related to their inherent biological activity in addition to the effects of their breakdown products. Many of beneficial health effects of these phytochemicals are considered to be based on their antioxidant activity, namely on their ability to scavenge free radicals and reactive oxygen species (ROS), as well as on their capacity to participate in complexation processes with macromolecules [158]. When analyzing the antioxidant efficacy of EA and its derivatives (taking into account the correlation of activity with the number of hydroxyl groups in the molecule [144, 198]), these compounds can be arranged in the following sequence (from left): ellagitannins, free form of EA, and EA conjugates [199].

The article "Ellagic Acid: A Review on Its Natural Sources, Chemical Stability, and Therapeutic Potential" was retracted in 2024. Reasons: signs of a paper mill; compromised peer review; unreliable results or conclusions.

Ellagitannins are also capable of exhibiting potent antimicrobial [200–203] and antiviral [204, 205], inhibiting mutagenicity of carcinogens, and stimulating host-mediated antitumor effects [6, 8, 94, 191, 193–195, 206, 207].

## 4. Degradation of Ellagic Acid and Ellagitannins in the Gastrointestinal Tract

In addition to the free form of EA, which enters the body with plant food, the major portion of this compound can arise in the digestive tract of humans and animals as a result of the hydrolytic degradation of ellagitannins present in foodstuffs. Therefore, EA content can be used to indirectly quantify ellagitannins present in plant foods and also as a biomarker of dietary bioavailability of ellagitannins [178, 208].

Studies on animal models and human volunteers consuming ellagitannin-rich food have shown that hydrolysis of ellagitannins and EA release occurs in the stomach and/or small intestine [209, 210]. Ester bonds in ellagitannins are relatively slowly hydrolyzed, resulting in prolonged gastrointestinal secretion of EA [211].

In the gastrointestinal tract, EA has a low bioavailability due to its hydrophobic moiety and very low water solubility and is only partly absorbed in the small intestine [121]. Unabsorbed EA molecules are further metabolized by intestinal microorganisms of the large intestine to form a series of metabolites known as urolithins (urolithins A–D) (Figure 2) [209, 212]. Urolithins are a subgroup of dibenzo[*b*,*d*]pyran-6-ones, which are formed by removing one of the lactone groups present in EA via lactonase/decarboxylase activity, followed by dehydroxylation reactions leading to the sequential removal of hydroxyl groups with the formation of urolithins D, C, A and B (tetrahydroxy-, trihydroxy-, dihydroxy-, and monohydroxy-dibenzopyran-6-one metabolites, respectively) [212]. These metabolites are absorbed into the bloodstream as their lipophilicity increases and can circulate throughout the body before being excreted in the urine [212–214].

In enterocytes and hepatocytes, urolithins can undergo biotransformation with the formation of a combination of urolithin metabolites [209]. The main metabolites of urolithins found in plasma and urine are their glucuronyl and sulfate conjugates [215]. The main ellagitannin metabolites that appear in urine and plasma are urolithin A and B glucuronide and sulfate, while the minor metabolites are urolithin C and isourolithin A glucuronide [128, 216–218].

The article "Ellagic Acid: A Review on Its Natural Sources, Chemical Stability, and Therapeutic Potential" was retracted in 2024. Reasons: signs of a paper mill; compromised peer review; unreliable results or conclusions.

Urolithins appear in plasma and urine within a few hours (5 hours or more) after ingestion of food containing ellagitannins, being detectable in plasma and urine within 48–72 hours in free and conjugated forms [212, 219, 220].

EA and urolithins can accumulate in the intestine and prostate [53, 221, 222]. After intraperitoneal and oral administration of synthesized urolithins to mice, the concentrations of these compounds reached higher levels in the prostate, colon, and intestine tissues compared with other organs [222].

It is considered that pathway of EA metabolism to urolithins is characteristic of mammals, since birds and insects that feed on food containing ellagitannins do not produce urolithins [215]. Ulaszewska et al. [218] point to the potential importance of urolithins as candidate biomarkers for assessing the consumption of certain food items, such as ellagitannin-rich berries (especially strawberries and raspberries) in humans.

The presence of urolithins has also been reported in ellagitannin-rich plants such as pomegranate leaves [223], in the fruit of water caltrop (*Trapa natans* L.) [224, 225], and in Nile tamarisk (*Tamarix senegalensis* DC.) flowers, which also contain EA and are known in Egyptian traditional medicine as antiseptic, antipyretic, and anti-inflammatory remedy [226]. Urolithins are also important constituents of shilajit used in Ayurvedic medicine [227].

Urolithins are biologically active compounds exhibiting strong antioxidant effects [178, 225, 228–230] and possessing potential anti-inflammatory [211, 231], chemopreventive [146], antiproliferative [35, 221], and neuroprotective [232, 233] properties.

## 5. Preclinical Pharmacological Activities of Ellagic Acid

EA is a polyphenol found in diverse fruits and nuts, which has been associated with a variety of health benefits, many of them related to oxidative stress [2, 211, 234–236]. Although it has been reported that EA has a low water solubility and poor bioavailability, many efforts have been performed to improve such conditions. Here, we will briefly describe the experimental data supporting the benefits of EA consumption in the prevention of oxidative stress and inflammation, its potential use as a treatment of different kinds of cancer, metabolic syndrome, as well as the protective potential of EA for liver, central nervous system (CNS), and skin related diseases (Figure 3).

The article "Ellagic Acid: A Review on Its Natural Sources, Chemical Stability, and Therapeutic Potential" was retracted in 2024. Reasons: signs of a paper mill; compromised peer review; unreliable results or conclusions.

### 5.1. Role of EA against Oxidative Stress

Along with ascorbic acid and *α*-tocopherol, EA is considered one of the major antioxidant molecules [237]. The chemical structure of EA, containing two lactones and four hydroxyl groups, enables scavenging a wide variety of ROS. Although at physiological pH and in aqueous solution EA can deactivate peroxyl radicals, hydroxyl radicals, nitrogen dioxide, and peroxynitrite [16, 238], better scavenging capacities have been computed for ROS compared to reactive nitrogen species [239]. EA is considered an unusual protector against oxidative stress, due to its predicted capacity to regenerate and not being reduced after its metabolism, enabling this polyphenolic compound to provide continuous protection even at low concentrations [16].

Ionic metals such as copper, iron, nickel, and cadmium are a potential source of oxidative stress, and EA is able to chelate these metals providing an additional protection mechanism against this condition [16, 240, 241]. The importance of these mechanisms was demonstrated by Ahmed et al. [242], where the consumption of EA (500 *μ*mol/kg body weight) by female Wistar rats, protected them against the cadmium-induced oxidative stress in the liver and kidney.

Oxidative stress can damage DNA, and the production of 8-oxo-2-deoxyguanosine is a typical marker of this process. This can lead to mutations and in consequence to cancer and other health conditions. It was shown that EA significantly decreases the amount of 8-oxo-2-deoxyguanosine produced after oxidative DNA damage [243], which correlates well with the capacity of EA to bind DNA, likely proving a protection mechanism against free radicals [244, 245]. Moreover, oxidative damage on DNA induced by dopamine/Cu^2+^ was alleviated by EA, even when doses as low as 1 *μ*M were used, reaching 50% of DNA decomposition inhibition [246].

EA is not only able to scavenge prooxidant agents, but also EA increases the expression/activity of antioxidant enzymes (superoxide dismutase, glutathione peroxidase, glutathione reductase, and catalase) in Dalton's lymphoma-bearing mice treated with this phenolic compound [247]. A similar regulation of the antioxidant enzymes and regulation of the Nrf2 redox sensitive transcription factor was observed in human dermal fibroblast, after UV-B light-induced oxidative stress and treatment with EA [18].

In the initiation and propagation of lipid peroxidation, hydroxyl and peroxyl radicals are involved. Low concentrations of EA (20 *μ*M) have proven effective suppressing lipid peroxidation induced by *γ*-radiation in microsomes [238]. Boyuk et al. [248] measured the levels of malondialdehyde (MDA), a product of lipid peroxidation, in rats after ischemia reperfusion, and observed lower levels of this marker in individuals treated with EA (85 mg/kg body weight), which presumably could be related to EA free radical scavenging effect.

The article "Ellagic Acid: A Review on Its Natural Sources, Chemical Stability, and Therapeutic Potential" was retracted in 2024. Reasons: signs of a paper mill; compromised peer review; unreliable results or conclusions.

### 5.2. Anti-inflammatory Effects of EA and Its Consequences in Associated Pathologies

There is a close relation between oxidative stress and inflammation [249]. As previously described, EA can provide protection against oxidative stress via due to its own chemical properties but also modulating the expression of enzymes involved in this process. Although these antioxidative properties could help to prevent inflammation, it has been demonstrated that EA has itself potent anti-inflammatory activities in cell cultures (*in vitro*) and *in vivo* [250].

Inflammation is a process that involves the activation or inhibition of a number of cytokinins such as interleukins (IL) and tumor necrosis factor- (TNF-) *α*, as well as transcription factors, e.g., interferon gamma (IFN-*γ*) and nuclear factor- (NF-) *κ*B. On the other hand, the expression of adhesion molecules in endothelial cells is recognized as an early step in inflammation and atherogenesis. This enables an interaction between the endothelium and immune cells [251]. In a study where human aortic cells were treated with EA (0.1-10 *μ*M), an inhibition of TNF-*α*-induced endothelial activation and expression of both vascular cell adhesion molecule- (VCAM-) 1 and intercellular cell adhesion molecule- (ICAM-) 1 was observed [83]. This suggests that EA has a high antiatherogenic potential and hence can provide protection against cardiovascular diseases (Figure 4). In a different study, the effects of EA supplementation were evaluated in human umbilical vein endothelial cells (HUVEC) treated with IL-1*β* to induce the expression of VCAM-1, ICAM-1, and E-selectin [252]. The application of EA (25-50 *μ*M) reduced the expression of VCAM-1 and E-selectin and significantly prevented the binding of monocytes to IL-1*β*-induced HUVEC, confirming the anti-inflammatory properties of EA and its potential role preventing atherosclerosis. Furthermore, this study demonstrated that EA was able to prevent the nuclear translocation of p50/p65 (both subunits of NF-*κ*B), which suggest that this polyphenolic compound avoids the expression of adhesion molecules at the transcriptional level. In this line, it has been shown that EA can modulate the expression of proinflammatory mediators *in vivo*. For instance, when EA was administrated (58.33 mg/kg body weight) to an adjuvant-induced arthritis mouse model, the serum levels of the proinflammatory cytokines IL-1*β*, TNF-*α*, and IL-17 were significantly reduced [253]. EA-mediated reduction in IL-17 (at the mRNA and protein level) was also observed in C57BL/6 J mice fed with 0.2% cup to induce oligodendrocytes depletion [254]. In this investigation, a high dose of EA (80 mg/kg body weight/day/i.p., 4 weeks) prevented brain damage via reduction of neuroinflammation and toxic effects of cup on mature oligodendrocytes, meaning that EA could be a suitable therapeutic agent for diseases such as multiple sclerosis.

The article "Ellagic Acid: A Review on Its Natural Sources, Chemical Stability, and Therapeutic Potential" was retracted in 2024. Reasons: signs of a paper mill; compromised peer review; unreliable results or conclusions.

### 5.3. Potential Chemopreventive and Therapeutic Uses of EA in Cancer

Several studies have provided evidence of the chemopreventive and therapeutic effects of EA either derived from the diet or administered via different matrices optimized to improve its bioavailability [235, 250]. Since oxidative stress causes multiple damages on DNA, inducing mutations in the protooncogenes and tumor suppressor genes, EA could be a potential agent to promote the antioxidant response and therefore overcome the carcinogenesis process. This was evaluated in Dalton's lymphoma-bearing mice treated with three different doses (40, 60, and 80 mg/kg body weight) of EA [247]. All doses of EA contributed efficiently to reduce the Protein C signaling (involved in cell proliferation and tumor growth) via NF-*κ*B and also improved the antioxidant defense. These effects could explain the cancer preventive role of EA.

*In vitro* studies where different cancer cell lines, including Caco-2, breast, and human prostatic cancer cells, were treated with EA (10-100 *μ*M) demonstrated the strong antiproliferative activity exerted by this polyphenolic compound [255]. The best antiproliferative effects were observed in Caco-2 cells, whereas breast cancer cells where the most resistant ones to EA application. Another study demonstrated that EA induces apoptosis on Caco-2 via the intrinsic pathway, implying mitochondrial release of cytochrome c and activation of caspases [53]. Furthermore, treatment of Caco-2 cells and HCT-116 cells with EA revealed expression changes in several genes involved in diverse cell functions such as proliferation, cell cycle, apoptosis, and angiogenesis [256, 257]. The anticancerous effect of EA against HCT-15 colon adenocarcinoma cells was recently evaluated by Umesalma et al. [258]. In this study, the EA treatment decreased the activity of alkaline phosphatase and lactate dehydrogenase, pointing to an antiproliferative and cytotoxic effect, respectively. Interestingly, EA increased the production of ROS, induced apoptosis, and decreased cell proliferation of HCT-15 cells, suggesting that it could act as an efficient agent against colon cancer. On the other hand, several investigations have focused on the prevention and therapy potential of AE on breast cancer. Among the effects of EA in MCF-7 cells (a model for breast cancer) are (1) prevention of cell proliferation and migration, (2) apoptosis induction, inhibition of angiogenesis, (3) inhibition of cell growth, and (4) decreased cell viability (Figure 5) [259]. In addition, PJ and three of its components (including EA) are inhibitory of metastatic processes in breast cancer and modulate the expression of genes related to cell migration, cell adhesion, and those that control chemotaxis [260]. Since a major limitation of EA as chemopreventive and therapeutic agent against cancer relies on its low bioavailability, many efforts have been directed towards improvements in this direction. For instance, nanoencapsulation of pomegranate polyphenols including EA and punicalagin resulted in efficient uptake by MCF-7 cells, and a 2- to 12-fold enhanced effect on growth inhibition, when compared to free polyphenols [261]. As important as breast cancer is prostate cancer, which is responsible for numerous deaths of men worldwide [262]. In early stages, prostate cancer can be treated with hormones, but over time, the cancer turns insensitive to hormones and becomes more aggressive and metastasizes [263]. EA along with luteolin and punicic acid were able to inhibit hormone independent and dependent growth of prostate cancer cells [264] but also proved to be effective preventing metastasis *in vivo* using mouse models [265]. In the same study, the combination of polyphenols was effective in preventing angiogenesis and inhibiting human endothelial cell tube formation, thus providing an effective alternative to inhibit prostate cancer progression and metastasis.

The article "Ellagic Acid: A Review on Its Natural Sources, Chemical Stability, and Therapeutic Potential" was retracted in 2024. Reasons: signs of a paper mill; compromised peer review; unreliable results or conclusions.

### 5.4. Positive Effects of EA on Glucose and Lipid Metabolism and Its Protective Effect on Organs

Elevated lipid and glucose levels, along with abdominal obesity, high blood pressure, and low high-density lipoprotein- (HDL-) cholesterol levels, are among the factors increasing the risks for heart disease, diabetes, and stroke and are considered the main features of metabolic syndrome. Oxidative stress contributes to the pathogenesis of type 2 diabetes and the concomitant diabetic vascular complications [266–268]. Among the positive effects of EA on glucose metabolism and diabetes in murine models are (a) reduction of glucose levels; (b) antioxidant, antiglycation, and ant-inflammatory effects; and (c) prevention of micro- and macrovascular diabetic complications [51]. In a recent study, free EA and EA nanoparticles were administrated to diabetic rats fed a high-fat diet. The results demonstrated that EA nanoparticles improved glucose levels and body weight for longer periods compared to regular EA [269]. Moreover, better results for EA nanoparticles were also observed on lipid profile markers, such as total cholesterol, triglycerides, low-density lipoprotein (LDL), and very-low-density lipoprotein (VLDL), and insulin production levels. Resistin is an adipocytokine considered to act as a link between obesity and type 2 diabetes. When EA was supplemented to a mouse model for obese type 2 diabetes fed a high-fat diet, improved serum lipid profile and hepatic steatosis were observed [270]. Furthermore, reduced serum resistin levels were found in adipose tissue, along with higher mRNA levels of genes that promote lipid oxidation, suggesting a possible mechanics to improve obesity-induced dyslipidemia.

The article "Ellagic Acid: A Review on Its Natural Sources, Chemical Stability, and Therapeutic Potential" was retracted in 2024. Reasons: signs of a paper mill; compromised peer review; unreliable results or conclusions.

Thanks to its efficient antioxidant capacity, EA exhibits promising activities as a potential organ protective agent *in vitro* and *in vivo*. For instance, some of the main neuroprotective effects of EA against different stressor compounds used in rat models are lower levels of DNA damage, IL downregulation, decreased lipid peroxidation, lower reactive species production and improvements in memory function, neuronal function, and antioxidant enzyme production [271]. Hepatoprotective effects have been attributed to EA since it improves the hepatic functions against toxic and pathological conditions, due to its antioxidant, antihepatotoxic, antisteatotic, anticholestatic, antifibrogenic, antihepatocarcinogenic, and antiviral properties [64]. Several experiments on murine models have shown that the molecular mechanisms of EA to exert its hepatoprotective role include the scavenging of free radicals, regulation of antioxidant enzymes, modulation of proinflammatory cytokines synthesis, the regulation of lipids synthesis, and degradation, among others (Figure 6) [64]. Interestingly, EA has potential antiviral properties against hepatitis B [272] and hepatitis C [273] virus, both able to lead in the long term to fibrosis, cirrhosis and hepatocellular carcinoma [274].

UV-B radiation induces of collagen breakdown and inflammation in skin cell [275, 276]. To test the potential protective effect of EA on keratinocytes and human dermal fibroblast, Bae et al. [84] exposed these cells to UV-B radiation and treated them with the phenolic compound (1-10 *μ*M). An attenuation of the UV-B damage in both types of cells was observed, along with a decrease in collagen degradation because of lower levels metalloproteinase production. Additionally, the same authors found that topical application of EA (10 *μ*M) protected hairless mice from skin wrinkle formation when they were exposed to UV-B. This positive response was associated with lower production of proinflammatory cytokines (IL-1*β* and IL-6) and mitigation of ICAM-1 expression. The use of EA as functional ingredient in cosmetic products has been proposed due to its antioxidant, skin-lightening, and sunscreen properties. In this line, efforts have been made to improve EA solubility and stability through the preparation of gold nanoparticles wrapped with chitosan to absorb EA [277]. Good and promising results were obtained when the above-mentioned properties were evaluated and highlight as well that the nanoparticles were produced according green chemistry principles.

The article "Ellagic Acid: A Review on Its Natural Sources, Chemical Stability, and Therapeutic Potential" was retracted in 2024. Reasons: signs of a paper mill; compromised peer review; unreliable results or conclusions.

## 6. Ellagic Acid in Clinical Trials

In this review, we included clinical trials that test the efficacy of EA in itself (Table 2). However, we also considered studies that evaluated primary EA sources, i.e., pomegranate (*P. granatum*). The reader should interpret those results considering that said primary sources contain other compounds besides EA. Thus, we cannot evaluate its effect directly. Also, where applicable, we focused on clinical/patient-centered endpoints and not surrogate endpoints.

### 6.1. Exercise Performance and Postexercise Recovery

A 2018 systematic review with eleven studies and 230 participants concluded that pomegranate supplementation might improve strength performance and endurance and accelerate postexercise recovery. PJ should contain at least one gram of polyphenols per 750 mL (recommended amount), taken at least one hour before exercise and within 48 hours after exercise. It is also most effective in resistance training in well-trained populations [278].

### 6.2. Cognitive Function

Liu et al. [279] performed a randomized clinical trial (RCT) that evaluated EA's efficacy on cognitive improvement in middle-aged men using the Wechsler Adult Intelligence Scale-Revised (WAIS-R) and Montreal Cognitive Assessment test (MoCA). Patients were randomly assigned to receive 50 mg EA or placebo daily for 12 weeks. While the EA arm obtained statistically significant higher scores in overweight men, there were no differences in patients with normal body mass index (BMI) [279]. However, the reader should interpret these results with caution. The average scores in each group are not present. Still, a rough estimate based on graphs hints that the difference between groups might not be clinically significant, as WAIS-R scores in both groups were within normal limits. More recent WAIS versions are preferred as a measurement scale [298]. Also, there is no fixed cut-off point for the MoCA test to understand if there was a clear difference in cognitive function between groups. Furthermore, twelve weeks is a relatively short time to consider significant cognition improvements.

The article "Ellagic Acid: A Review on Its Natural Sources, Chemical Stability, and Therapeutic Potential" was retracted in 2024. Reasons: signs of a paper mill; compromised peer review; unreliable results or conclusions.

An additional RCT with a 12-month follow-up assessed PJ's memory effects (8 oz daily, 29 mg EA) on middle-aged and older adults. The authors used the Brief Visuospatial Memory Test-Revised (BVMT-R) and Buschke Selective Reminding Test (SRT) as primary outcome instruments. In general, there were no significant differences between the intervention and placebo groups. Nevertheless, visual learning remained the same since baseline in patients that drank PJ while it declined in the placebo group. Overweight or obese status did not interact with the treatment effect [299].

### 6.3. Skin Conditions

A systematic review focused on the efficacy of natural ingredients in managing hyperpigmentation disorders found two RCTs that evaluated EA use [280]. One study assessed using a preparation of 0.5% EA and 0.1% salicylic acid and compared it to 4% hydroquinone in patients with hyperpigmentation and dark spots. After 12 weeks of treatment, the EA and salicylic compound performed similarly to the benchmark agent. Additionally, the sensory analysis seems to give the novel combination an edge. The second study compared the efficacy of 1% arbutin, synthetic 1% EA, and synthetic 1% EA combined with plant extracts containing natural EA in treating 30 patients with melasma. All three treatment groups showed significant improvement after treatment. However, both studies have limitations. The first study did not consider EA in itself but as a combination with salicylic acid [281]. The second study did not compare the extracts independently [282].

Henning et al. [283] randomized 74 women to receive 8 oz of PJ (23 mg EA), 1000 mg of pomegranate extract (same dose of EA as juice), or placebo for twelve weeks. They found that either the liquid or the placebo significantly increased the minimal erythema dose. Therefore, it may lead to increased UV damage protection [283].

*Platycarya strobilacea* Siebold & Zucc. extract, mainly containing EA, also seems to have antiwrinkle activity, increasing the expression of type I collagen mRNA and more significant visual differences compared to placebo [284].

### 6.4. Insulin Resistance and Diabetes

A 2020 systematic review on the hypoglycemic effect of pomegranate by Virgen-Carrillo et al. [300] revealed that the evidence's methodology is heterogeneous, including study design and intervention characteristics. The studies' patients varied widely in clinical features: healthy, obese, diabetic people, metabolic syndrome, cardiovascular pathologies, and women with polycystic ovarian syndrome [300].

Of the twelve studies considered in this review, two report a significant reduction in glucose levels after PJ ingestion, one after 3 hours, and the second after six weeks after exposure [285, 286]. However, these are pretest-posttest studies; there is no placebo or standard care group used as a comparison. Additionally, these studies on patients with type 2 diabetes do not report the use of hypoglycemic drugs. The studies that indicate that used hypoglycemic drugs did not find a positive effect with PJ [289, 301, 302]. Amor et al. [51] also suggest that the impact of EA on glucose management is inconclusive.

The article "Ellagic Acid: A Review on Its Natural Sources, Chemical Stability, and Therapeutic Potential" was retracted in 2024. Reasons: signs of a paper mill; compromised peer review; unreliable results or conclusions.

### 6.5. Weight and Body Composition

“Functional foods” such as pomegranate have been considered a tool in managing overweight and obesity. Yet, Gheflati et al. [287] report on their systematic review that there was no significant effect of pomegranate consumption on body weight, BMI, waist circumference, or body fat percentage.

### 6.6. Cardiovascular Disease Risk Factors

#### 6.6.1. Carotid Artery Intima-Media Thickness (CAIMT)

This is a surrogate marker of atherosclerosis and is considered a strong predictor for stroke and myocardial infarction. Aviram et al. [288] investigated whether the CAIMT changes by consuming PJ in patients with asymptomatic carotid artery stenosis. There were a total of 19 patients in the study; 10 of them received the intervention. After one year of treatment, there was a statistically significant decrease in CAIMT (*p* < 0.01). The authors do not specify the mean CAIMT nor confidence intervals, but from the graphs, we can estimate that the CAIMT reduces from 1.5 mm to 1.1 mm, approximately. The mean CAIMT and the standard deviation were, however, reported for patients in the placebo group. There was a statistically significant increase, from1.52 ± 0.03 to1.65 mm + 0.04 mm (*p* < 0.01) after a year of follow-up. However, there is no report of head-to-head comparisons between groups. Additionally, a subgroup of patients received the treatment for three years, and there is no data about the final mean CAIMT for those patients [288].

Davidson et al. [291] evaluated PJ's effects on CAIMT in patients at moderate risk for coronary heart disease. After 18 months of treatment, participants in the intervention group (*n* = 146) showed no significant difference in mean CAIMT (0.79 vs. 0.80, *p* = 0.168) or the overall CAIMT progression rate between PJ and control treatments (0.005 ± 0.004 mm, *p* = 0.654) [291].

#### 6.6.2. Peak Systolic Velocity (PSV) and End-Diastolic Velocity (EDV)

In [288], there was a statistically significant decrease in mean PSV and EDV of both left and right carotid arteries after PJ consumption (*p* < 0.01) after one year of treatment. There is no report of exact mean values or confidence intervals for either the control or intervention group either before or after treatment; there is only a graph that roughly hints at the mean changes in the PJ group. Therefore, there are no data on comparisons between groups. Again, as with CAIMT, they do not report data on patients that received treatment for three years [288].

The article "Ellagic Acid: A Review on Its Natural Sources, Chemical Stability, and Therapeutic Potential" was retracted in 2024. Reasons: signs of a paper mill; compromised peer review; unreliable results or conclusions.

#### 6.6.3. Stress-Induced Ischemia

In [289], patients with stable coronary heart disease were randomly assigned to a PJ group or a placebo group. Participants underwent electrocardiographic-gated myocardial perfusion single-photon emission computed tomographic technetium-99 m tetrofosmin scintigraphy at rest and during stress at baseline and three months after. There was a significant reduction (*p* < 0.05) in stress-induced ischemia in the PJ arm (summed difference score:−0.8 ± 2.7) compared to the placebo group (SDS1.2 ± 3.1) [289].

#### 6.6.4. Blood Pressure

The antioxidant activity of pomegranate and some evidence in animals that show it can inhibit the angiotensin-converting enzyme has made pomegranate an attractive compound for managing hypertension. However, Gbinigie et al. [303] indicate that there is conflicting evidence to support these benefits. The authors included eight RCTs in the review, and three studies reported significant reductions in systolic blood pressure. Two reported a significant decrease in diastolic blood pressure in patients receiving pomegranate. The writers expressed their concerns about the quality of the study design and the studies' short duration [291].

A different systematic review concluded significant blood pressure differences between those receiving pomegranate and controls [290]. However, there are some differences between these reviews. Although the second summary of the evidence includes an additional study that shows a significant decrease in systolic blood pressure, it does not consider a study in hemodialysis patients that shows no differences. Also, an RCT by Sohrab et al. [301], not included in [290], does not preestablish blood pressure as an outcome. Therefore, it should not be considered. Something concerning is that the second review recognizes two studies as evidence of a statistical difference between those receiving pomegranate and controls, when, in fact, those studies report no difference. For this reason, this review inclines to agree with [303].

#### 6.6.5. Lipid Profile

Although polyphenols seem to provide antioxidant activity and positively affect cardiovascular risk factors, it might not effectively manage lipid levels. A 2016 systematic review focused on twelve RCTs evaluating pomegranate consumption's benefits on the lipid profile found no significant effect of pomegranate consumption on plasma concentrations of cholesterol, LDL-C, HDL-C, or triglycerides [293]. These results are supported by a 2020 systematic review focused on the same subject [292].

The article "Ellagic Acid: A Review on Its Natural Sources, Chemical Stability, and Therapeutic Potential" was retracted in 2024. Reasons: signs of a paper mill; compromised peer review; unreliable results or conclusions.

### 6.7. Osteoarthritis

A randomized controlled trial without a placebo published in 2016 examined PJ's effects on clinical signs, inflammation, and antioxidant status in patients with knee osteoarthritis. After six weeks of treatment, patients who drank PJ had a statistically significant decrease in WOMAC stiffness and physical function scores (fewer symptoms) than baseline. However, there were no differences between the intervention and control groups [294].

### 6.8. Fatigue and Insomnia

A small nonrandomized controlled trial without a placebo evaluated the benefits of Robuvit® (extract from wood of *Quercus robur* L. containing ellagitannins roburin A-E, EA and gallic acid) on fatigue and insomnia. Patients chose which group to enter, and the Fatigue Severity Scale assessed fatigue while the Regensburg Insomnia Scale and Pittsburgh Sleep Quality Index assessed insomnia. Though there was a statistically significant improvement in fatigue and insomnia questionnaire scores after eight weeks of taking Robuvit®, the study does not report comparisons between the intervention and control group [295].

### 6.9. Prostate Cancer

Falsaperla et al. [296] evaluated EA effects as an adjuvant therapy for chemotherapeutic treatment in men with hormone-refractory prostate cancer (HRPC). Patients receiving EA had less risk of developing neutropenia than patients receiving chemotherapy alone (33.3% vs. 74.9%, respectively, *p* < 0.05). Gastrointestinal side effects seemed lower in the intervention group, although results were not statistically significant. Other positive outcomes in the EA group, though statistically nonsignificant, were as follows: PSA reduction, cases with complete response to chemotherapy, pain control, and quality of life. There were no differences in overall survival and progression-free survival between groups [296]. It is worth mentioning that the chemotherapy used was vinorelbine and estramustine phosphate, and other medications are more effective in this type of cancer, i.e., docetaxel [304]. Therefore, studies using first-line therapies should be considered when conducting new clinical trials.

### 6.10. Human Fertility

A 2014 Danish RCT evaluated the effects of tablets' consumption with *P. granatum* extract and *A. galanga* powder's standardized content on the total number of motile spermatozoa (TMSC) and sperm morphology defined by strict criteria in adult men with reduced semen quality. After three months of treatment, there was a statistically significant increase in TMSC after three months of the intervention (*p* = 0.026). However, the difference in follow-up TMSC between groups was not statistically significant. There were no differences in sperm morphology after treatment. The study size was small (*n* = 66), which might be one reason why no statistically significant differences were found. There is a need for larger RCTs, preferably evaluating EA with no combination [297].

The article "Ellagic Acid: A Review on Its Natural Sources, Chemical Stability, and Therapeutic Potential" was retracted in 2024. Reasons: signs of a paper mill; compromised peer review; unreliable results or conclusions.

## 7. Conclusions

Known as a naturally occurring bioactive and pharmacologically active polyphenolic compound, EA possesses a remarkable broad spectrum of therapeutic activities in addition to pharmacological potentials to treat numerous diseases and ailments. Findings from this review indicate EA may be involved in regulating a spectrum of cellular signaling pathways to prevent, mitigate, or slow down the progression of chronic disorders, including cardiovascular and neurodegenerative diseases, diabetes, and cancer. In addition, there is also evidence of a positive therapeutic effect of the combination of EA with other antioxidants, known for their multiple bioactivities and therapeutic potential. Due to a wide range of biological effects of EA, edible plants containing this phytochemical and its hydrolyzable derivatives, mainly ellagitannins, are a valuable source of EA for humans and belong to functional foods that promote health and may reduce the risk of disease. EA is also currently used in the pharmaceutical and cosmetics industries; consequently, various plant species are now being studied for EA content in order to find novel sources of EA in human nutrition, as well as sources of raw materials for the preparation of functional nutritional supplements and nutraceuticals. In modern medicine, natural substances represent an unlimited source of active molecules whose medical applications may increase in the near future. For this reason, it is very important to clarify the molecular mechanisms underlying the observed beneficial activities. Currently for EA, as for many other natural compounds, it is not completely clear whether for some observed beneficial effects, such as antineoplastic activity, a transcriptional action is necessary or whether they are mainly related to epigenetic action. Therefore, a large number of nutraceutical and therapeutic interventions can be designed, considering the possible mechanisms of this active agent and its precursors.

## Figures and Tables

**Figure 1:** Formation of ellagic acid upon hydrolysis of ellagitannin [184].

**Figure 2:** Absorption and metabolism routes of ellagitannins and ellagic acid.

**Figure 3:** Biological effects of ellagic acid (EA).

The article "Ellagic Acid: A Review on Its Natural Sources, Chemical Stability, and Therapeutic Potential" was retracted in 2024. Reasons: signs of a paper mill; compromised peer review; unreliable results or conclusions.

**Figure 4:** Anti-inflammatory effects of ellagic acid (EA) and its consequences in cardiovascular diseases.

**Figure 5:** Potential chemopreventive and therapeutic uses of ellagic acid (EA) in cancer.

**Figure 6:** Hepatoprotective role of ellagic acid (EA).

**Table 1:** The content of ellagic acid in fruits and seeds of various food plants (taking into account the total level of ellagic acid after hydrolysis of ellagitannins).

Plant species	Common name	EA content (mg/kg)	References
*Carya illinoinensis* (Wangenh.) K.Koch	Pecan	330^a^	[135]
*Castanea sativa* Mill.	Sweet chestnut	340-500^a^ (leaf) 1410-3210^a^ (bur) 240-900^a^ (outer shell) 800-1370^a^ (inner shell)	[149]
*Fragaria* × *ananassa* (Weston) Duchesne ex Rozier	Strawberry	630^a^ 683–853^b^	[135, 145]
*Hippophae rhamnoides* L.	Sea buckthorn	10^b^	[145]
*Juglans nigra* L.	Black walnut	590^a^	[135]
*Myrciaria dubia* (Kunth) McVaugh	Camu-camu	258.5^a^ (pulp) 5657^a^ (flour)	[139]
*Psidium guajava* L.	Guava	57.2–306^a^	[150]
*Punica granatum* L.	Pomegranate	700^a^ (arils) 38700^a^ (mesocarp)	[140]
*Rosa rugosa* Thunb.	Rose hip	1096^b^	[145]
*Rubus arcticus* L.	Arctic bramble (arctic raspberry)	3900^b^	[151]
*Rubus chamaemorus* L.	Cloudberry	3151^b^	[145]
*Rubus idaeus* L.	Raspberry	1500^a^ 2637–3309^b^	[135, 145]
*Rubus ursinus* Cham. & Schltdl.	Blackberry	1500^a^	[135]
*Rubus ursinus* × *Rubus idaeus*	Boysenberry	4960^a^ 1684^a^	[125, 148]
*Terminalia ferdinandiana* Exell	Gubinge (Kakadu plum)	8796^a^	[125]
*Vaccinium* spp.	Cranberry	120^a^	[135]
*Vitis rotundifolia* Michx.	Muscadine grape	360–912^b^	[12]

^a^Dry weight base. ^b^Fresh weight base.

**Table 2:** Ellagic acid in clinical trials.

Clinical trials	Results	References
Exercise performance	Improves strength performance and endurance and accelerates postexercise recovery	[278]
Cognitive function	Cognitive improvement in overweight men; improves visual learning	[279]
Skin conditions	Induce improvement in patients with hyperpigmentation and dark spots	[280]
	Patients with melasma showed significant improvement after treatment	[281, 282]
	Lead to increased UV damage protection	[283]
	Have antiwrinkle activity, increasing the expression of type I collagen mRNA	[284]
Insulin resistance and diabetes	Induce reduction in blood glucose levels	[285, 286]
Weight and body composition	No significant effect on body weight, body mass index, waist circumference, or body fat percentage	[287]
Cardiovascular disease risk factors	Decrease carotid artery intima-media thickness; decrease in mean peak systolic velocity and end-diastolic velocity of carotid arteries	[288]
	Reduction in stress-induced ischemia	[289]
	Significant reductions in systolic and diastolic blood pressure	[290, 291]
	No effect on plasma concentrations of cholesterol, LDL-C, HDL-C, or triglycerides	[292, 293]
Osteoarthritis	Significant decrease in WOMAC stiffness and physical function scores	[294]
Fatigue, insomnia	Improvement in fatigue and insomnia questionnaire scores	[295]
Prostate cancer	Ellagic acid effects as adjuvant therapy for chemotherapeutic treatment: less risk of developing neutropenia than patients receiving chemotherapy alone; PSA reduction; reduction gastrointestinal side effects	[296]
Human fertility	Increase in total number of motile spermatozoa	[297]

The article "Ellagic Acid: A Review on Its Natural Sources, Chemical Stability, and Therapeutic Potential" was retracted in 2024. Reasons: signs of a paper mill; compromised peer review; unreliable results or conclusions.

## Data Availability

The data supporting this review are from previously reported studies and datasets, which have been cited. The processed data are available from the corresponding author upon request.
